# Design of Sponsored Search Auction Mechanism for Federated Learning Advertising Platform

This article has been retracted.

**DOI:** 10.1155/2022/5787491

**Published:** 2022-04-07

**Authors:** Hong Jiang, Tianxu Cui, Kaiwen Yang

**Affiliations:** ^1^School of Management, Shenzhen Polytechnic, Shenzhen 518055, China; ^2^School of Information, Beijing Wuzi University, Beijing 101149, China

## Abstract

Federated learning has demonstrated strong capabilities in terms of addressing concerns related to data islands and privacy protection. However, in real application scenarios, participants in federated learning have difficulty matching. For example, two companies distributed in different regions do not know that the other party also needs federated learning in the case of information asymmetry. Therefore, it is difficult to build alliances. To enable suppliers and consumers to find one or more federated learning objects that are relatively satisfactory in a short time, this paper considers the idea of establishing a federated learning advertising platform, where data transactions need to consider privacy protection. A sponsored search auction mechanism design method is introduced to solve the problem of ranking the presentation order of participant advertisements. Due to the potential malicious bidding problem, which occurs when using the classic sponsored search auction mechanism under the federated learning scenario, this paper proposes a novel federated sponsored search auction mechanism based on the Myerson theorem, improving upon the ranking index used in the classic sponsored search auction mechanism. A large number of experimental results on a simulation data set show that our proposed method can fairly select and rank the data providers participating in the bidding. Compared with other benchmark mechanisms, the malicious bidding rate is significantly decreased. In the long run, the proposed mechanism can encourage more data providers to participate in the federated learning platform, thus continuously promoting the establishment of a federated learning ecosystem.

## 1. Introduction

In recent years, with the application of artificial intelligence in all walks of life [1], data privacy protection has become increasingly valued by individuals and organizations. On the one hand, people are unwilling to share data that contain personal information any more, due to the potential risk of privacy leakage. On the other hand, regulatory agencies in various regions and countries have also issued a series of policies and regulations to protect the security of private data. For example, the General Data Protection Regulation (GDPR) [2], officially implemented by the European Union in May 2018, puts forward the most stringent requirements for data privacy and security. This is currently the most comprehensive and widely used privacy protection law in the world. In China, the “Implementation Regulations of the Consumer Protection Law of the People's Republic of China”, promulgated in August 2016, applies to most companies that deal with consumer data, forcing companies to take responsibility for their obligations to protect consumer personal information.

Federated Learning (FL) has demonstrated strong capabilities in addressing data islands and privacy protection. Within the past few years, federated learning has developed rapidly, in terms of algorithms, frameworks, platforms, and applications, since Google first proposed the concept in 2016. To incentivize high-quality data providers to contribute their data to the federation, researchers have designed different incentive mechanisms. However, in the real environment, data are stored at the edge nodes of various institutions.

For a certain federated learning task, some uncertain information exists in the following aspects:

1. Which data providers have the willingness to contribute data? What is the sample size that they can provide? What are the features? How much will it cost?
2. Which data users have a demand for data? What types of data do the data users need? What is the quantity demand? How much will they pay for it?

To enable suppliers and consumers to find one or more FL objects that are relatively satisfactory in the shortest time, it is necessary to provide a Federated Learning advertising platform. The data provider, on the supply side, can publish a brief introduction about their data on the advertising platform. Data users, on the demand side, can also find their intended customers on the platform. After matching, the data provider and the data user will train a machine learning model together using federated learning. As shown in Figure 1, the federated learning advertising platform provides advertising slots and charges advertising fees. Data providers post advertisements on the platform and pay the fees. Data users then browse the advertisements, and send out invitations to intended customers for federated learning.

Generally speaking, some data providers want their ads to appear in the most attractive slot: the first place in the result page. However, the slots for displaying advertisements are limited. Therefore, for each search, the FL advertising platform faces the problem of matching advertisements with slots. In addition, the FL advertising platform also needs to determine the price that each data provider needs to pay. Data providers naturally prefer eye-catching slots. Therefore, to allocate a slot and determine the corresponding bid, the FL advertising platform needs a ranking system. There are an increasing number of data providers who want to post ads on the platform, but the number of available ad slots remains the same. To solve this problem, we can use an auction mechanism. These auctions are called Sponsored Search Auctions [3]. In a typical sponsored search auction, the data provider is invited to bid on the keywords, that is, for each click on the advertisement, the advertiser expresses the maximum amount they are willing to pay. This is usually referred to as cost-per-click (CPC). According to the bid submitted by the advertisers for a specific keyword, the search engine selects a set of advertisements and determines their presentation order. The actual price of the search engine also depends on the bid submitted by the customers. However, the sponsored search auction mechanism (GFP, GSP, VCG) mentioned above is not directly applicable to the scenario of federated learning as, if the bid is the only factor considered in the allocations of data providers, it may lead to malicious bidding and the emergence of monopoly issues. Many data providers which have noisy data in their data set will make higher bids to occupy the top slots on the advertising platform. Obviously, this is irresponsible to both the suppliers and consumers. In the long run, the advertising platform will suffer serious losses.

To resolve the above problems, we propose a new mechanism, called Federated Sponsored Search Auction Mechanism (FSSA), which is specific to the scenario of federated learning. Based on the bids, this paper also adds an index to reflect the average contribution of data providers in their previous federated learning scenarios, and assign certain weights to these two indices. Thus, a new ranking index is formally defined, ranking scores, which is more in line with the scenario of federated learning. The core idea is to consider both the bid and contribution to rank the data providers, such that some data providers whose data quality is poor but have strong economic strength can gain higher ad slots in the advertising platform; in the same way, some participants who lack money but who have better data quality can also rank highly on the advertising platform. Most importantly, this mechanism curbs the monopoly problem, to a certain extent, and secures the platform's long-term prosperity. Extensive experimental results on a simulation data set show that the FSSA can filter and rank the data providers participating in the bidding. Compared with the classic sponsored search auction mechanism, the malicious bidding rate can be significantly decreased, effectively avoiding the problem of inconsistency between the bid and the actual contribution ability.

Our contributions can be summarized as follows:

- In response to the difficulty of matching data providers and data users in federated learning, we first propose the idea of establishing an FL advertising platform. This platform can help both the suppliers and consumers to find a relatively satisfactory federated learning object in the shortest time. Furthermore, a new ranking mechanism is proposed to solve the problem of ranking advertisement slots.
- For the classic sponsored search auction mechanism, only bids are considered for the ranking, thus leading to malicious bids. We propose a new ranking index—ranking scores—which considers both the bids and historical average contributions of federated learning participants. To a certain extent, the problem of malicious bids can be avoided.
- We conduct extensive experiments on different simulation data sets to verify the effectiveness of our proposed method. The experimental results show that our method can effectively rank data providers. Compared with the classic sponsored search auction mechanism, the rate of malicious bidding is significantly decreased.

The remainder of this paper is arranged as follows: We summarize the related literature in Section 2. The method and results are detailed in Section 3. In Section 4, we conclude the paper and discuss some prospects for future work. To the best of our knowledge, this is the first time that the theory of sponsored search auctions has been applied to a federated learning scenario. The factors which we consider are not only the bids of data providers but also a comprehensive survey of their contributions. A novel mechanism is proposed to ensure that the data providers of the FL advertising platform are treated fairly, as well as to encourage more data providers to participate in the federated learning platform, in order to promote the establishment of the federated learning ecology.

## 2. Literature Review

We review the related literature from the following three aspects: Federated learning, mechanism design, and sponsored search auctions.

### 2.1. Federated Learning

Federated learning is a distributed machine learning framework [4, 5], which aims to solve the problems of user privacy and data islands which occur in the process of machine learning. Without data transmission, this method can train a machine learning model through using data from various devices. Since Google first proposed federated learning in 2016 [6], it has been favored by many technology companies, and many specialized research teams have been established. Not only have they achieved a lot of research results in frameworks and algorithms but also have actively explored and advanced the business landing applications of federated learning. Yang et al. [7] have expanded the concept and application of federated learning. According to the distribution features of data islands, federated learning can be divided into three types: horizontal federated learning, vertical federated learning, and federated transfer learning.

Recent research into federated learning has mainly focused on privacy protection and incentive mechanisms. To prevent the leakage of private data during gradient and parameter sharing in federated learning, researchers have applied traditional privacy protection techniques to federated learning, mainly divided into the following aspects: Secure multi-party computing [8–10], homomorphic encryption [11, 12], and differential privacy [13–15]. Some studies have begun to use the immutability of blockchain technology [16, 17] for privacy protection in federated learning. In terms of incentive mechanism design, Cong et al. [18] have established a research framework for the design and reasoning of federated learning incentive mechanisms, and proposed a precise definition of the FML incentive mechanism design problem. They divided this big problem into demand and supply-side problems for research and design. Zeng et al. [19] conducted a comprehensive research review on the design of federated learning incentive mechanisms. They showed that the Federated Shapley value retains the desirable properties of the canonical Shapley value; it can be calculated without incurring additional communication costs, and it can also capture the influence of the participation order on data value. Different from the above works, Wei et al. [20] have proposed the concept of contribution index—a new metric based on Shapley value—which is suitable for evaluating the contribution of each data provider in the joint model of joint learning training. To solve the problem related to the large amount of calculations needed for the contribution index, they proposed two gradient-based methods. In addition, many scholars have introduced auction theory into the design process of the reward mechanism of federated learning. Kim et al. [21] have studied the incentive mechanism and privacy protection of federated learning from the perspective of mechanism design. Jiao et al. [22] have proposed an auction-based market model to encourage data owners to participate in joint learning, and designed two auction mechanisms for the federated learning platform to maximize the social welfare of the federated learning service market. In this paper, when defining the ranking scores of the FL advertising platform, we use a federated learning participant contribution index, which was defined and used by Wei et al. [20]. The contribution of each participant in federated learning can be measured fairly, to a certain extent, which, to some degree, represents the quality of the data held by the participant.

### 2.2. Mechanism Design

Hurwicz [23] first proposed the concept of mechanism design in the 1960s. He defined mechanism design as systems that can communicate with each other. It is the process of assigning results to participants, based on pre-made rules and information received in each round. In 1961, Vickrey published a paper on the second-price sealed-bid auction (i.e., a Vickrey Auction) [24], which was a milestone in the field of mechanism design. Three papers on incomplete information game theory, published by Harsanyi in the 1960s [25, 27], laid a solid foundation for mechanism design. Hurwicz introduced the concept of incentive compatibility into the field of mechanism design in 1972, thus opening up a period of rapid development in mechanism design [28]. Soon after, Clarke [29] and Groves [30] extended the Vickrey mechanism to a more general quasilinear environment, and developed a more general incentive compatibility. In the 1970s, thanks to the joint efforts of a group of outstanding scholars, such as Gibbard [31] and Maskin [32], mechanism design made great progress in the revelation principle and implementation theory. As time progressed, mechanism design has been applied to many different disciplines, such as auctions, design of markets and trading institutions [33, 34], social choice theory [35], computer science [3], and so on.

### 2.3. Sponsored Search Auctions

The auction is the core content of mechanism design research, and sponsored search auctions have been a hotspot in the field of computer science over the past decade [36]. For traditional revenue optimization, Myerson [37] solved the single-term problem in the Bayesian–Nash equilibrium environment. Krysta et al. [38] have studied the multi-unit optimal auction. Since the first sponsored search auction was initiated in 1997, a series of auction mechanisms have been proposed, such as Overture's Generalized First Price (GFP) auction [39] and Google's Generalized Second Price (GSP), which has caused sponsored search auctions to become an important source of income for online platforms. Due to the inauthenticity of GSP, Garg et al. [40], based on the previous work, modeled the sponsored search auction on the Internet as a mechanism design problem, and designed a novel optimal auction mechanism (OPT), which can maximize the expected benefits of search engines while achieving Bayesian incentive compatibility and individual rationality. Lahaie et al. [41] have proposed another idea of compressing GSP parameters to increase income. Ostrovsky et al. [42] applied these works and studied the impact on Yahoo using auctions with the best reserve price. Zhang et al. [43] proposed an online reverse auction scheme for cloud computing service allocation based on Vickrey–Clarke–Groves (VCG) mechanism and online algorithm (OA), which can help cloud users and providers to build workflow applications in the cloud computing environment. This analytical approach has important implications for measuring the performance of the proposed algorithm without assuming the distribution of cloud provider bids.

As for the trade-off between different goals, some related studies can be found in the literature. Sundararajan et al. [44] have considered a convex combination of income and welfare to improve the forecast. Li et al. [45] constructed an integrated system with a mixed arrangement of advertising and organic items, and determined the best trade-off between instant income and user experience. In addition, for different settings and actual requirements, they extended the proposed optimal truthful allocation mechanism to meet these realistic conditions. With the help of real data, they verified the advantages of the proposed mechanism over the classic Myerson optimal advertising mechanism. Lian et al. [46] have optimized the advertising pruning of sponsored search based on reinforcement learning. This is the first time that reinforcement learning technology has been used to address this problem. More importantly, it has been successfully implemented in Baidu's sponsored search system, and online long-term A/B tests have shown a significant increment in revenue.

## 3. Method and Results

### 3.1. Preliminary Knowledge and definition

#### 3.1.1. Typical Service Process of FL Advertising Platform

**Step 1 .**

As shown in Figure 2, the federated learning client enters keywords to search for a certain learning task on the advertising platform.

**Step 2 .**

After receiving the keywords, the federated learning advertising platform ranks the *n* bids *b*^(*j*)^ associated with the keywords of data providers using the ranking allocation rules, which are set in advance. After ranking, *m* data providers are selected, who are then ranked according to their ranking scores *r*^(*j*)^.

**Step 3 .**

The customer browses the data set information provided by data providers on the advertising platform, selecting one or more data providers that they are satisfied with. Then, the client sends them an invitation for federated learning, and matches them according to their intentions to form a federated learning alliance.

**Step 4 .**

The paired data providers and customers conduct federated learning as an alliance, and the benefits are allocated according to the profit allocation rules set in advance (not the focus of this paper, and will not be repeated). After completing federated learning, the final contribution index c^(*j*)^ of each participant is the output.

**Step 5 .**

The FL advertising platform charges the data providers for advertising fees *p*_*j*_, in accordance with the payment rules.

#### 3.1.2. Mechanism Design Environment Setting

In this paper, we propose an ad-sponsored search platform for federated learning. Aiming to solve the matching problem of participants in the federated learning scenario, our goal is to find a set of optimal allocation rules and payment rules to maximize the benefits of the FL advertising platform and meet certain constraints on the design of sponsored search auction mechanisms. Our assumptions were as follows:

(1) There are *n* data owners *j* who are interested in a certain federated learning task, where *J*={1,2,…, *n*} represents a set of data providers. In addition, the alliance has *m* advertising slots *k*, where data providers can place their own basic data information (e.g., sample size, characteristics, data quality, and data cost), where *K*={1,  2,…*m*} denotes the set of these advertising slots.
(2) *α*_*jk*_ is the probability that a data user clicks when the data provider *j* is in the *k*^*th*^ advertisement slot, where slot 1 represents the highest slot (the most prominent slot). We assume that *α*_*jk*_ satisfies the following conditions:
  (1) $$\begin{array}{c} 1\geq \alpha_{j1}\geq \alpha_{j2}1\geq \cdots \geq \alpha_{jm}\geq 0\;\forall j\in J\forall k\in K. \end{array}$$
(3) For any federated learning task, each data provider *j* who is interested in this task makes a bid *b*^(*j*)^ ≥ 0, where *b*^(*j*)^ depends on their economic behavior in the real market environment, with a certain degree of randomness.
(4) Each data provider knows exactly how much value they can get when any data user clicks on their advertisement once. We assume that this value has nothing to do with the ad position, and this value only depends on whether the data user clicks on its ad. The data provider *j* does not know the value that other data providers get from one click of the data user. Formally, we assume that the value that data provider *j* gets from each click of a data user is *v*^(*j*)^. The parameter *v*^(*j*)^ is called the valuation of data provider *j*, and the set of possible valuations of this provider is denoted as *V*^(*j*)^.
(5) Each data provider *j* has a federated learning contribution index *c*^(*j*)^, which measures the quality of their own data. It is worth noting that the contribution degree represents the true contribution ability of the data provider; it has nothing to do with the bid and can truly reflect the value of the data owned by the data provider. This contribution can be calculated through a variety of mechanisms. In this paper, we use the method proposed by Wei et al. [20] to calculate the contribution index based on the Shapley value.
(6) Each data provider *j* is rational and intelligent, which means they pursue the maximum expected value of the utility function *u*^(*j*)^, which we define later.

According to the above model assumptions, the sponsored search auction problem of the FL advertising platform can be accurately described as follows. Whenever the FL advertising platform receives the keywords of this federated learning task, it uses the bid profile *b*=(*b*^(1)^, *b*^(2)^,…*b*^(*j*)^ …, *b*^(*n*)^) and contribution index profile *c*=(*c*^(1)^, *c*^(2)^,…*c*^(*j*)^ …, *c*^(*n*)^) to determine: (1) Which data providers can win the slots to present their advertisements, as well as the order in which their advertisements are presented and (2) when data users click on their advertisements, the amount of money each data provider should pay to the platform. The former is the allocation rule, and the latter is the payment rule.

We define the problem environment of the sponsored search mechanism design in a typical FL advertising platform as follows:

(i) Result set X : A result of the federated advertising sponsored search auction is a vector *x*=(*y*_*jk*_, *p*_*j*_), ∀*j* ∈ *J*; ∀*k* ∈ *K*, where *y*_*jk*_ is the probability that data provider *j* is assigned to slot *k*, and *p*_*j*_ is the cost-per-click paid by the data provider to the FL advertising platform. Therefore, the feasible result set can be expressed as:
  (2) $$\begin{array}{c} \text{X}=\left\{\left(y_{jk},p_{j}\right)|y_{jk}\in \left\{0,1\right\};\sum_{j=1}^{n}y_{jk}\leq 1;\sum_{k=1}^{m}y_{jk}\leq 1\text{;}p_{j}\geq 0,\forall j\in J;\forall k\in K\right\}. \end{array}$$
(ii) Utility function *u*^(*j*)^(•): Given a result *x*, the utility function of data provider *j* can be expressed as:
  (3) $$\begin{array}{c} u^{\left(j\right)}\left(x\left(r\right),b^{\left(j\right)}\right)=\left(\sum_{k=1}^{m}y_{jk}\alpha_{jk}\right)\left(b^{\left(j\right)}-p_{j}\right). \end{array}$$
(iii) Social surplus function *W*: In this case, the utility of all data providers constitutes the social surplus function of the entire alliance. This is expressed as:
  (4) $$\begin{array}{c} W=\sum_{j=1}^{n}u^{\left(j\right)}\left(x\left(r\right),b^{\left(j\right)}\right),\;\forall j\in J. \end{array}$$

For convenience, we summarize the defined symbols and their meanings in Table 1.

### 3.2. Federated Learning Advertising Platform Sponsored Search Auction Mechanism Design

We define the sponsored search mechanism design problem of a typical federated learning advertising platform as follows:

Let *b*=(*b*^(1)^, *b*^(2)^,…*b*^(*j*)^ …, *b*^(*n*)^) and *c*=(*c*^(1)^, *c*^(2)^,…*c*^(*j*)^ …, *c*^(*n*)^) be the bid profile and contribution index profile of data provider *j*, respectively. Let *b*^(−*j*)^ and *c*^(−*j*)^ denote the bid and contribution index profile of all other participants except for data provider*j*, respectively. As the bid profile is affected by multiple factors in actual production and the real world, it has a certain degree of randomness, which may lead to the problem of malicious bidding. For this reason, we propose a new ranking index, *r*=(*r*^(1)^, *r*^(2)^,…, *r*^(*n*)^), which is composed of the bid profile *b*^(*j*)^ and the contribution index profile *c*^(*j*)^, that is,

(5) $$\begin{array}{c} r^{\left(j\right)}\left(b^{\left(j\right)}\right)\underline{\underline{\text{def}}}\left(\beta \varphi^{\left(j\right)}\left(b^{\left(j\right)}\right)+\left(1-\beta \right)c^{\left(j\right)}\left(\varphi^{\left(j\right)}\left(b^{\left(j\right)}\right)\right)\right), \end{array}$$

where *c*^(*j*)^(•) is contribution index function. In Ref. [20], Wei et al. proposed an effective federated learning contribution index calculation method based on the Shapley value. We also use a similar method to calculate the contribution index:

(6) $$\begin{array}{c} c^{\left(j\right)}\left(\varphi^{\left(j\right)}\left(b^{\left(j\right)}\right)\right)=\sum_{S\subseteq J\backslash \left\{j\right\}}\frac{\left|S\right|!\left(\left|J\right|-\left|S\right|-1\right)!}{\left|J\right|!}\left\{v^{\prime }\left(S\cup \left\{j\right\}\right)-v^{\prime }\left(S\right)\right\}, \end{array}$$

where *S* is a subset of *J*,

(7) $$\begin{array}{c} v^{\prime }\left(S\cup \left\{j\right\}\right)=\sum_{j^{\prime }\in \left(S\cup \left\{j\right\}\right)}\varphi^{\left(j^{\prime }\right)}\left(b^{\left(j^{\prime }\right)}\right)=\sum_{j^{\prime }\in \left(S\cup \left\{j\right\}\right)}\left(b^{\left(j^{\prime }\right)}-\frac{1-F^{\left(j^{\prime }\right)}\left(b^{\left(j^{\prime }\right)}\right)}{f^{\left(j^{\prime }\right)}\left(b^{\left(j^{\prime }\right)}\right)}\right),\\ v^{\prime }\left(s\right)=\sum_{j^{\prime }\in S}\varphi^{\left(j^{\prime }\right)}\left(b^{\left(j^{\prime }\right)}\right)=\sum_{j^{\prime }\in S}\left(b^{\left(j^{\prime }\right)}-\frac{1-F^{\left(j^{\prime }\right)}\left(b^{\left(j^{\prime }\right)}\right)}{f^{\left(j^{\prime }\right)}\left(b^{\left(j^{\prime }\right)}\right)}\right), \end{array}$$

where *φ*^(*j*′)^ represents the virtual value of data provider *j*′,

(8) $$\begin{array}{c} \varphi^{\left(j^{\prime }\right)}\left(b^{\left(j^{\prime }\right)}\right)=b^{\left(j^{\prime }\right)}-\frac{1-F^{\left(j^{\prime }\right)}\left(b^{\left(j^{\prime }\right)}\right)}{f^{\left(j^{\prime }\right)}\left(b^{\left(j^{\prime }\right)}\right)}, \end{array}$$

where *F*^(*j*′)^(*b*^(*j*′)^) is the cumulative distribution of its bid, and the corresponding probability density function is *f*^(*j*′)^(*b*^(*j*′)^). These need to satisfy the following assumptions:

**Assumption 1 .**

(Distribution of bid). For each data provider *j*, we assume that their bid *b*^(*j*)^ is independently—but not necessarily identically—drawn from a known cumulative distribution *F*^(*j*)^(*b*^(*j*)^), where the corresponding probability density function is *f*^(*j*)^(*b*^(*j*)^).

**Assumption 2 .**

(Monotonicity of virtual value). For each data provider *j*, we assume that the cumulative distribution of its bid *F*^(*j*)^(*b*^(*j*)^) satisfies the regular condition; thus, the virtual value *φ*^(*j*)^(*b*^(*j*)^) is monotone nondecreasing.

Note that *β* ∈ [0,  1] is a variable parameter indicating the proportion of virtual value *φ*^(*j*)^(•) to the contribution index *c*^(*j*)^(•). We provide its calculation method later.

After the FL advertising platform receives the participant's bids, the platform calculates the ranking score *r*, and then ranks the participants according to their ranking score. Therefore, a mechanism *X*=(*x*(*r*), *p*(*r*)) consists of two rules, the allocation rule *x*(*r*) and the payment rule *p*(*r*); more specifically, *x*(*r*)=(*x*_1_(*r*), *x*_2_(*r*),…, *x*_*n*_(*r*)) and *p*(*r*)=(*p*_1_(*r*), *p*_2_(*r*),…, *p*_*n*_(*r*)), where *x*_*j*_(*r*)=∑_*k*=1_^*m*^*y*_*jk*_*α*_*jk*_.∀*jεJ*; ∀*kεK*, *y*_*jk*_ is the probability that the data provider *j* is assigned to the *k*^*th*^ slot, and *p*_*j*_ is the cost-per-click that the data provider pays to the FL advertising platform. Therefore, the feasible result set, *X*, can be expressed as:

(9) $$\begin{array}{c} \text{X}=\left\{\left(y_{jk},p_{j}\right)|vy_{jk}\in \left\{0,1\right\};\sum_{j=1}^{n}y_{jk}\leq 1;\sum_{k=1}^{m}y_{jk}\leq 1;p_{j}\geq 0,\forall j\in J;\forall k\in K\right\}. \end{array}$$

It is worth noting that random results are also included in the above result set, which means that random mechanisms are also part of the mechanism space.

Given the result *x*, the utility function *u*^(*j*)^(•) of the data provider *j* can be expressed as:

(10) $$\begin{array}{c} u^{\left(j\right)}\left(x\left(r\right),b^{\left(j\right)}\right)=\left(\sum_{k=1}^{m}y_{jk}\alpha_{jk}\right)\left(b^{\left(j\right)}-p_{j}\right). \end{array}$$

In the FL advertising platform system, to ensure that data providers always have the willingness to auction, we require that the utility of data provider *j* should not be less than zero, that is, we demand that each data provider satisfies individual rationality. We define this as follows:

**Definition 1 .**

(Individual Rationality).

(11) $$\begin{array}{c} u^{\left(j\right)}\left(x\left(r\right),b^{\left(j\right)}\right)\geq 0,\;\forall j\in J;\;\forall k\in K. \end{array}$$

In addition, to avoid malicious bidding by data providers, we impose Bayesian Incentive Compatibility (BIC) constraints on the designed mechanism:

**Definition 2 .**

(Bayesian Incentive Compatibility).

(12) $$\begin{array}{c} u^{\left(j\right)}\left(x\left(r\right),v^{\left(j\right)}\right)\geq u^{\left(j\right)}\left(x\left(r\right),b^{\left(j\right)}\right),\;\forall j\in J. \end{array}$$

If and only if a mechanism meets the conditions of IR and BIC, we call it a feasible mechanism. Myerson's theorem gives equivalent expressions for IR and BIC. Similarly, we can also design a mechanism with IR and BIC on the FL advertising platform, as shown below:

**Lemma 1 .**

(Myerson theorem) [37]. If and only if a mechanism satisfies IR and BIC, for any advertisement item from data provider *j* and bids of other items *b*^(−*j*)^, the allocation rule *y*_*j*_(*b*^(*j*)^, *b*^(−*j*)^), is monotone nondecreasing on *b*^(*j*)^, and the payment rule is as follows:

(13) $$\begin{array}{c} p_{j}\left(b\right)=\left\{\begin{array}{cc} b^{\left(j\right)}-\;\frac{\int_{0}^{b^{\left(j\right)}}y_{j}\left(x^{\left(j\right)},b^{\left(-j\right)}\right)dx^{\left(j\right)}}{y_{j}\left(b\right)}, & y_{j}\left(b\right)\neq 0.\\ 0, & else. \end{array}\right. \end{array}$$

In summary, we have the following mechanisms.

(1) Allocation rules
  (14) $$\begin{array}{c} y_{jk}\left(b\right)=\left\{\begin{array}{cc} 1, & \text{if }r^{\left(j\right)}\left(b^{\left(j\right)}\right)\text{is }k^{th}\text{ highest ranking score, }k\in K,\\ 0, & else. \end{array}\right. \end{array}$$
(2) Payment rules
  (15) $$\begin{array}{c} p_{j}\left(b\right)=\left\{\begin{array}{cc} b^{\left(j\right)}-\;\frac{\int_{0}^{b^{\left(j\right)}}y_{j}\left(x^{\left(j\right)},b^{\left(-j\right)}\right)dx^{\left(j\right)}}{y_{j}\left(b\right)}, & y_{j}\left(b\right)\neq 0.\\ 0, & else. \end{array}\right. \end{array}$$
Now, we give the calculation method for the coefficient *β*. Specifically, in such a mechanism, we require that the total social utility should be maximized, that is, the total social surplus *W* is maximized under certain constraints, making the malicious bidding rate *μ* (defined later) lower than that in classic sponsored search auction mechanisms.
  (16) $$\begin{array}{c} \max\text{W.} \end{array}$$
  (17) $$\begin{array}{c} s.t.\;\left\{\begin{array}{c} u^{\left(j\right)}\left(x\left(r\right),b^{\left(j\right)}\right)\geq 0;\\ u^{\left(j\right)}\left(x\left(r\right),v^{\left(j\right)}\right)\geq u^{\left(j\right)}\left(x\left(r\right),b^{\left(j\right)}\right);\\ \sum_{k=1}^{m}y_{jk}\leq 1;\\ \sum_{j=1}^{n}y_{jk}\leq 1;\\ 0\leq y_{jk}\leq 1;\\ p_{j}\geq 0;\\ \forall j\in J;\\ \forall k\in K. \end{array}\right. \end{array}$$

For the above constrained programming, we use the Lagrange multiplier method to solve the equation. The Lagrange function can be expressed as follows:

(18) $$\begin{array}{c} L=W+\left(\lambda \overset{n}{\underset{j=1}{\sum }}u^{\left(j\right)}\left(x\left(r\right),b^{\left(j\right)}\right)+\overset{n}{\underset{j=1}{\sum }}\left(u^{\left(j\right)}\left(x\left(r\right),v^{\left(j\right)}\right)-u^{\left(j\right)}\left(x\left(r\right),b^{\left(j\right)}\right)\right)+\overset{n}{\underset{j=1}{\sum }}\left(1-\overset{m}{\underset{k=1}{\sum }}y_{jk}\right)+\overset{m}{\underset{k=1}{\sum }}\left(1-\overset{n}{\underset{j=1}{\sum }}y_{jk}\right)+\overset{n}{\underset{j=1}{\sum }}\overset{m}{\underset{k=1}{\sum }}\left(1-y_{jk}\right)+\overset{n}{\underset{j=1}{\sum }}\overset{m}{\underset{k=1}{\sum }}y_{jk}+\overset{n}{\underset{j=1}{\sum }}p_{j}\right), \end{array}$$

where *λ* is the Lagrange multiplier, *λ*=(*λ*_1_, *λ*_2_,…, *λ*_4*n*+*m*+2*mn*_).

For ease of the descriptions, we use Ω to represent all the constraints. Thus, the Lagrange function can be expressed as follows:

(19) $$\begin{array}{c} L=W+\lambda \cdot \Omega , \end{array}$$

where Ω ≥ 0.

As *W* is a linear function of *y*, the constraints are also linear in *y*, and the result set is a convex set, and the constrained program in (16) and (17) consists of convex optimization. We can obtain the optimal value of the coefficient *β* in the equation of ranking score by Lemma 2.

**Lemma 2 .**

(Optimal estimation of coefficient) [45]. The constrained program with constraints given in (17) is equivalent to the unconstrained programming with coefficient *β*^*∗*^ and, when the optimal Lagrange multiplier is *λ*^*∗*^, the coefficient can be expressed as *β*^*∗*^=1/(||*λ*^*∗*^||+1) We obtain ‖*λ*^*∗*^‖ by Algorithm 1. Then, we can obtain *β*^*∗*^.

Algorithm 1 shows the detailed process for calculating the ranking score *r*^(*j*)^ of each data provider*j*. Specifically, lines 1–12 are the calculation of coefficient *β*, while lines 13 and 14 are the calculation of the ranking score *r*^(*j*)^.

**Theorem 1 .**

(FSSA). When a federated learning advertising platform satisfies Assumptions 1 and 2 under the conditions of Definitions 1 and 2, and takes Equation (5) as the ranking score, an optimal mechanism can be obtained.

**Proof**

When Assumptions 1 and 2 are satisfied, we can construct a ranking score based on contribution index and virtual value with the help of Equations (6) and equation (8), that is, Equation (5). As it is under the conditions of Definitions 1 and 2, Lemma 1 holds, and the calculation expressions of allocation rules and payment rules can be obtained. As the linear program constructed under the above conditions satisfies convexity, Lemma 2 holds, and the optimal estimate of the coefficients in the ranking score can be obtained. Q.E.D.

### 3.3. Simulation Experiment Design

To evaluate the performance of our proposed federated learning advertising platform sponsored search auction mechanism (FSSA) algorithm, we carried out many simulation experiments using *Python*. To verify whether the malicious bidding rate of FSSA had changed, we compared it with four classic mechanisms based on bid *b_i_* ranking, under the same simulation data set and experimental environment settings. The experiment was run on a Windows 10 desktop with 32 GB main memory, an Intel Xeon E5-2690 v3 @2.60 GHz(X2) CPU with 12 cores and 24 threads, and an NVIDIA GeForce GTX1060 6 GB graphics card.

#### 3.3.1. Data Set

In a real market environment, a data provider's bid is related to many factors, and the data provider may not report its bid *b*^(*j*)^ in a truthful way. Therefore, in this experiment, we assumed that each bid *b*^(*j*)^ obeys a uniform distribution, that is, *b*^(*j*)^ ~ *U*(0,1). Moreover, as the number of data providers and the number of advertising slots cannot be determined, we divided it into two situations to conduct separate experiments: (1) When *n* > *m*, assume that the number of data providers *n* is 8, and the number of ad slots *m* is 5, 6, or 7. The method of setting the click-through rate obeys the following principle: the click-through rate increases at equal intervals from 0.1 to 0.9, according to the number of ad slots (e.g., when *m*  = 5, the click probability *α*_*jk*_ of each advertising spot, from bottom to top, is from 0.1 to 0.9, having the same interval of 0.2 increases successively) and (2) when *n* ≤ *m*, assume that the number of data providers *n* is 5, and the number of ad slots is *m* and the click probability *α*_*jk*_ are the same as when *n* > *m*.

Algorithm 2 shows the detailed process for generating the training data set. Specifically, line 1 is the process of generating all possible ranking results set. As for each sample in the training data set, lines 3–17 show its generation process. Lines 18–20 show the process of generating a label for each training data sample, initializing the set {*r*^(*j*)^} to set {*r*_order_^(*j*)^} first, then ranking the elements in it in the descending order, using *r*_order_=(*r*_order_^(1)^, *r*_order_^(2)^,…, *r*_order_^(*j*)^,…, *r*_order_^(*n*)^) ∈ {list_*l*_*|l*=1,2,…, (min(*m*, *n*))!} to represent the ranking result. Finally, *r*_order_ is matched in the set {list_*l*_}, and the index of the matched *list*_*l*_ is taken as the label of the training data sample.

#### 3.3.2. Comparison Algorithm

We compared the malicious bidding rate of the proposed method with those of three classic sponsored search auction algorithms, which have been summarized by Narahari et al. in Ref. [3]. Due to space limitations, we do not review these algorithms in detail; instead, brief summaries are provided in the following.

GFP. This algorithm is the generalized first price auction mechanism. Under this mechanism, the *m* advertising positions are allocated to advertisers in the descending order, according to their bids.

GSP. This algorithm is the generalized second-price auction mechanism, which is adapted from the generalized first price auction mechanism. Due to the instability of the generalized first price, the entire system has low allocation efficiency; thus, GSP was proposed. This mechanism is completely consistent with the GFP allocation rules, but changes its payment rules. The participant who gets slot 1 pays the bid of the participant who wins slot 2, and so on.

VCG. This algorithm is the abbreviation of the Vickery–Clark–Groves mechanism, which is the most widely used mechanism in the field of mechanism design. In a quasilinear environment, the VCG mechanism not only has allocation efficiency but also incentive compatibility.

#### 3.3.3. Evaluation Metrics

To evaluate whether our proposed algorithm can effectively reduce the probability of malicious bidding problems or not, we defined a new evaluation index, the malicious bidding rate *μ*, which represents the cumulative number of malicious bidding events happening in *N* bidding scenarios.

(20) $$\begin{array}{c} \mu \;\underline{\underline{\text{def}}}\;\frac{1}{N}\overset{N}{\underset{i=1}{\sum }}M, \end{array}$$

where *M* represents a malicious bidding event. We define the distance between the result of the bid *b* or the ranking score *r* and the benchmark ranking *c* as the similarity *d*. If the similarity *d* is not 0, it indicates that a malicious bidding event *M* has happened, that is,

(21) $$\begin{array}{c} d\left(r_{\left(\cdot \right)},r_{\left(c\right)}\right)\underline{\underline{\text{def}}}\left\{\begin{array}{cc} \frac{1}{\text{score}\left(r_{\left(\cdot \right)},r_{\left(c\right)}\right)}, & \text{if score}\left(r_{\left(\cdot \right)},r_{\left(c\right)}\right)\neq 0,\\ +\infty , & \text{else,} \end{array}\right. \end{array}$$

where *r*_(·)_ represents the result of ranking by bid *b* or ranking score *r*; *r*_(*c*)_ represents the result of ranking by the contribution index *c*, which we call benchmark ranking; and score(*r*_(·)_, *r*_(*c*)_) represents the matching score between the ranking results. That is, for two sequences with the same length of *m*, starting from the first slot, if the *k*^*th*^ slot of *r*_(·)_ and *r*_(*c*)_ is the same, then the match of this slot is successful, and 1 point is counted; otherwise, 0 points are counted. Formally, we define the rank score as score $\text{score}\left(r_{\left(\cdot \right)},r_{\left(c\right)}\right)\underline{\underline{\text{def}}}\sum_{k=1}^{m}Match\left(r_{\left(\cdot \right)},r_{\left(c\right)}\right)$, where Match(*r*_(·)_, *r*_(*c*)_) represents the matching situation, which is:

(22) $$\begin{array}{c} \text{Match}\left(r_{\left(\cdot \right)},r_{\left(c\right)}\right)\underline{\underline{\text{def}}}\left\{\begin{array}{cc} 1, & \text{if }r_{\left(\cdot \right)}^{\left(k\right)}\;=\;r_{\left(c\right)}^{\left(k\right)}\\ 0, & \text{else,} \end{array},\;\forall k\in K.\right. \end{array}$$

Algorithm 3 shows the calculation process for the malicious bidding rate. In lines 1–7, we use Equation (22) to calculate the matching score and, in line 8, we use Equation (21) to calculate the similarity. Finally, we use Equation (20) to calculate the evaluation index malicious bidding rate *μ* in lines 9 and 10.

#### 3.3.4. Experimental Setup

In this paper, a convolutional neural network (CNN) model was used for training. Algorithm 4 shows the training process of the convolutional neural network (CNN) model, using the training data set and label set generated in Algorithm 2. Lines 1–3 show the initialization of the model parameters and the setting of the learning rate, while Lines 4–10 show the process of obtaining the optimal parameters of the neural network model through the backward propagation algorithm. Specifically, the model consists of two convolution layers and three fully connected layers. The output of each hidden layer is activated by the ReLU activation function, the dropout is set to 0.5. The backward propagation algorithm is used to solve the parameters, the optimizer is set to Adam, the loss function is set to sparse categorical crossentropy, and the learning rate is set to 0.001. The training batch size is set to 124, and the number of iterations is 200 rounds.

#### 3.3.5. Analysis of Results

As shown in Figure 3, the experimental results under different simulation experimental data sets confirmed that the performance of the FSSA mechanism proposed in this paper was better than that of the other benchmark mechanisms. This further proves the effectiveness and robustness of the FSSA mechanism for the ranking of the advertising slots in federated learning advertising platforms.

Specifically, when *n* ≤ *m* (i.e., *n*=5), from the horizontal perspective, *m* continues to increase. The accuracy of the four mechanisms showed little change. In this case, the number of participants was always less than the number of advertisements, so the participants were always fully allocated, and the complexity of the model changes mainly depend on min(*n*, *m*). Therefore, even if the number of advertising slots continues to increase, the accuracy of the model does not change much, and the model is relatively stable.

When *n* > *m* (i.e., *n*=8), from a horizontal perspective, with the continuous increase of *m*, the accuracy of the four mechanisms gradually decreased, and the speed of convergence also decreased. In this case, the number of participants was always greater than the number of advertisements, so there was the situation where there were remaining participants. The complexity of the model mainly depends on min(*n*, *m*). Therefore, with the continuous increase of *m*, the allocation rules that need to be considered are more complicated and the model complexity is high. In the end, the model converges slowly and the accuracy of the convergence is also reduced, in accordance with the actual situation.

For each case of *m*, with *m* is fixed, vertical comparison between *n*=5 and *n*=8 indicated that, when *n*=5, the number of participants is less than the number of advertising slots, and the advertising slots cannot be fully allocated. Compared with *n*=8, the latter had a richer allocation and a higher allocation efficiency, thus facilitating model convergence.

In Table 2, our testing accuracy of the model in different situations is shown. It can be seen that, no matter the situation, the testing accuracy of our proposed FSSA mechanism was higher than that of the benchmark.

As can be seen from Figure 4, when *n*=5, that is, participants were always less than the number of advertisements. With the increase of *m*, the accuracy of the four mechanisms showed little change, and this is because the remaining advertising space is always sufficient. For each participant, they are not sensitive to the dynamic changes of allocation rules or payment rules in the process of competition. Therefore, the learning degree of the model to the data features contained in the sample data tensor tends to be saturated. And, in this scenario, the testing accuracy of our proposed FSSA mechanism was higher than others. This means that FSSA can still learn the data distribution law relatively deeply when the data features are not obvious, so as to estimate the model parameters more accurately.

As can be seen from Figure 5, when *n*=8, that is, participants were always more than the number of advertisements. With the continuous increase of *m*, the testing accuracy of various mechanisms varies. And, in this scenario, there were remaining participants, and the complexity of the model mainly depends on min(*n*, *m*). Due to the fierce competition, the data tensor contains rich features, but it is also easy to cause the phenomenon of over fitting of model parameters, which makes the generalization ability of the model insufficient. In this case, GFP mechanism and GSP mechanism are difficult to deal with such problems, while VCG mechanism and FSSA mechanism alleviate the over fitting phenomenon on the premise of ensuring relatively high accuracy, and FSSA mechanism can still maintain relatively high testing accuracy. Thus, the feasibility and stability of the model are trustworthy.

We summarize the malicious bidding rates in different situations in Table 3. It can be seen, from the table, that the malicious bidding rate under our proposed FSSA mechanism was as low as 0.01016. Compared with the classic sponsored search auction mechanisms, the malicious bidding rate was greatly decreased under the same conditions, effectively reducing the probability of malicious bidding in the auction process for advertising slots on the Federated Learning advertising platform.

In addition, it can be seen, from Figure 6, that when *n* = 5, *m* increased, as all participants were allocated, and they had no motivation to lie. Therefore, the trend of the malicious bidding rate for the four mechanisms was not obvious. Within the same group of *m* and *n*, the malicious bidding rate under the conditions of GFP mechanism and GSP mechanism is relatively high. Therefore, it can be seen that the response ability of these two mechanisms to the phenomenon of malicious bidding is insufficient. In contrast, VCG mechanism reduces the malicious bidding rate to about 0.077, which is relatively obvious. Even so, the malicious bidding rate of our proposed FSSA mechanism was still far lower than other benchmark mechanisms, and it is always lower than 0.04. As shown in the figure, this mechanism has a significant effect on reducing the malicious bidding rate.

However, Figure 7 shows that, at *n* = 8, due to the surplus of participants, participants had greater motivation to lie. Therefore, when *m* increase linearly, the rate of malicious bidding also gradually increased; however, that of the proposed mechanism was still lower than those of the other benchmark mechanisms, in line with our expectations. Moreover, when we compare the experimental results shown in Figure 7 with those shown in Figure 6, we find that when *m* takes the same value, that is, when the same number of advertisements are supplied, the competition among participants is fierce, that is, as shown in Figure 7, the response ability of GFP, GSP, and VCG to malicious bidding is weakened, and only FSSA has not received any negative impact. Compared with the experimental results shown in Figure 6, its response ability to malicious bidding rate is more significant, and the malicious bidding rate is further reduced.

In summary, compared with other benchmark sponsored search auction mechanisms, our proposed FSSA mechanism can effectively curb the generation of malicious bidding in the process of sponsored search auctions for federated learning advertising slots without imposing incentive-compatible constraints, which still allows for the social resources to be fully allocated.

## 4. Conclusions

In this paper, we proposed a novel Federated Sponsored Search Auction Mechanism (FSSA) for the scenario of federated learning. Based on the original bidding, the average contribution index of the data providers in their previous federated learning scenarios is considered, and a certain weight is assigned to them. A new ranking index is formally defined, that we call ranking scores, which make the proposed mechanism more in line with the scenario of federated learning. We conducted a large number of experiments on different simulation data sets to verify the effectiveness of our proposed method. The experimental results demonstrated that our method can rank data providers fairly. Compared with classic sponsored search auction mechanisms, the malicious bidding rate was reduced significantly through the use of the proposed mechanism. The social resources were effectively allocated, and the establishment of the federated learning ecology was promoted.

However, when studying slot allocation in an FL advertising platform, we only considered the situation where there are a small amount of data providers and advertising slots. When the number of participants continues to increase, the stability of the model will decrease and the generalization ability of the model needs to be improved. In addition, due to the experimental cost and the requirements of data privacy protection regulations, we did not obtain a real experimental data set and only conducted our experiments on a simulated experimental data set. Our future work will focus on optimizing the parameters in order to improve the generalization ability of the used neural network models as well as to obtain real experimental data.

## Figures and Tables

**Figure 1:** Schematic diagram of the Federated Learning Advertising Platform.

**Figure 2:** Schematic diagram of the advertising space of the FL advertising platform.

**Figure 3:** Training accuracy of different mechanisms in various situations.

**Figure 4:** Testing accuracy of different mechanisms at *n* = 5.

**Figure 5:** Testing accuracy of different mechanisms at *n* = 8.

**Figure 6:** Malicious bidding rate under different mechanisms at *n* = 5.

**Figure 7:** Malicious bidding rate under different mechanisms at *n* = 8.

**Algorithm 1:** Calculation of the ranking score.*r*^(*j*)^.

**Algorithm 2:** Training data set generation.

**Algorithm 3:** Calculation of the malicious bidding rate*μ*.

**Algorithm 4:** CNN Training.

**Table 1:** List of mathematical symbols and their definitions.

Symbol	Meaning
*j*	Index of the data provider
*k*	Index of the advertising slot
*α*_*jk*_	Probability that the data user clicks the *k*^*th*^ ad slot
*b* ^(*j*)^	Bid from data provider *j*
*v* ^(*j*)^	Valuation from data provider *j*
*c* ^(*j*)^	FL contribution index of data provider *j*
*r* ^(*j*)^	Ranking score of data provider *j*
*x*=(*y*_*jk*_, *p*_*j*_)	Result set
*u* ^(*j*)^(•)	Utility function of data provider *j*
*W*	Social surplus function

**Table 2:** Testing accuracy of different mechanisms in various situations.

(n,m)	GFP	GSP	VCG	FSSA
(5,5)	0.76434	0.76551	0.77223	0.78366
(5,6)	0.76509	0.76601	0.77206	0.78949
(5,7)	0.76584	0.76706	0.77270	079063
(8,5)	0.76634	0.76449	0.79811	0.80984
(8,6)	0.76676	0.76427	0.79907	0.80877
(8,7)	0.76716	0.76494	0.78411	0.80143

**Table 3:** Malicious bidding rate of different mechanisms in various situations.

(n,m)	GFP	GSP	VCG	FSSA
(5,5)	0.12566	0.11449	0.07777	0.03634
(5,6)	0.12491	0.11399	0.07794	0.03051
(5,7)	012416	0.11294	0.07730	0.02937
(8,5)	0.22366	0.21551	0.15199	0.01016
(8,6)	0.22324	0.21573	0.15093	0.01123
(8,7)	0.22284	0.21506	0.16589	0.01857

## Data Availability

The data used to support the results of this study are currently in the privacy protection stage and can be obtained from the corresponding author upon request 6 months after the article is published.
